The article "Effects and Satisfaction of Comfort Nursing plus Psychological Nursing in the Clinical Nursing of Neurology Patients: A Comparative Study" was retracted in 2023. Reasons: unreliable results or conclusions; concerns about the data; concerns about the peer review; concerns about the citations.

# Effects and Satisfaction of Comfort Nursing plus Psychological Nursing in the Clinical Nursing of Neurology Patients: A Comparative Study

**DOI:** 10.1155/2022/8013787

**Published:** 2022-05-25

**Authors:** Lihua Zhang, Wei Zhang, Yuping Jiang, Kaifeng Yao

**Affiliations:** Department of Neurology, Nantong First People's Hospital, Nantong, Jiangsu, China

## Abstract

**Objective:**

To explore the effects and satisfaction of comfort nursing plus psychological nursing in the clinical nursing of neurology patients.

**Methods:**

In this prospective study, 90 neurology patients admitted to our hospital from January 2019 to January 2020 were recruited and randomized into a control group and an experimental group with 45 cases in each group. The control group received routine care, and the experimental group received comfort care plus psychological care. The comfort scores and nursing satisfaction of the two groups were compared. The Hospital Anxiety and Depression Scale (HAD) was used to assess the emotional state of patients before and after the intervention. The Exercise of Self-care Agency Scale (ESCA) was used to assess the patient's self-care ability after the intervention.

**Results:**

The comfort scores of the experimental group were higher than those of the control group (*P* < 0.05). The experimental group showed significantly higher satisfaction than the control group (*P* < 0.05). Patients in the experimental group had lower HAD scores after intervention than those in the control group (*P* < 0.05). After the intervention, the experimental group had higher ESCA scores and a higher Barthel index than the control group (*P* < 0.05).

**Conclusion:**

Comfort nursing plus psychological care improves nursing satisfaction and self-care ability of neurology patients and relieves their negative emotions.

## 1. Introduction

With the development of medical technology and the improvement of living standards, people's demand for neurological care is increasing [1, 2]. Conventional nursing fails to meet the nursing needs of patients and may further result in nurse-patient disputes [2, 3]. In addition, patients in the *Department of Neurology* are vulnerable to negative emotions, and the absence of effective psychological care is associated with compromised quality of life and self-care abilities. Clinically, comfort nursing plus psychological care contributes to avoiding nurse-patient dispute lieving patients' negative emotions and reducing adverse events [4–6], which facilitates the establishment of a harmonious nurse-patient relationship. Patients in the neurology department mostly suffer from consciousness disorders, mental abnormalities, and sensory, motor and cognitive impairment, and their conditions change rapidly and are predisposed to adverse events, which may lead to low patient satisfaction and more nurse-patient disputes. Thus, effective nursing management is of great significance in neurology care. To further investigate the application effect and satisfaction of comfortable nursing plus psychological nursing in the clinical nursing of neurology patients, 90 neurology patients admitted to our hospital from January 2019 to January 2020 were recruited.

## 2. Materials and Methods

### 2.1. Participants

In this prospective study, ninety neurology patients admitted to our hospital from January 2019 to January 2020 were recruited and randomized into a control group and an experimental group, with 45 cases in each group. The research was approved by the Ethics Committee of the Nantong First People's Hospital, and the ethics approval number is 2018-11-15.

### 2.2. Inclusion Criteria

Patients who were first admitted to the neurology department; without mental illness or confusion; who provided written informed consent were included.

### 2.3. Exclusion Criteria

Patients with severe immune system diseases; with cognitive disorders; and with severe organic diseases were excluded.

## 3. Methods

Patients in the control group received routine nursing care, including basic nursing, health education, medication guidance, diet guidance, and condition monitoring.

The experimental group received comfort nursing plus psychological nursing. (1) A nursing team was established and the nursing staff received professional training in comfort nursing and psychological nursing to improve their nursing quality. (2) A nursing plan was formulated for neurology patients according to their actual conditions. (3) The patients were given health education about the relevant factors and precautions of the disease to strengthen their treatment confidence and compliance. (4) An adverse event management protocol was established for the analysis of adverse events during nursing. (5) A comfortable hospitalization environment was provided for the patients. (6) Night treatment was performed when the patients were awake to avoid interference with sleeping, and patients were given a foot bath before bed. (7) The pain of the patients was regularly assessed. Drug analgesia was used for severe pain if necessary, and nondrug analgesia was used for mild pain relief. (8) The patients were actively communicated to evaluate their mental state. Psychological counseling was provided to help patients relieve their psychological pressures. (9) The patients' needs were timely fulfilled, and appropriate encouragement and guidance were provided to facilitate them maintain a positive attitude.

Patients with symptoms of wind-phlegm blockage were given traditional Chinese medicine preparations. Patients with hemiplegia were treated with acupuncture application at the acupoints of Quchi, Hegu, Zusanli, Shousanli, Waiguan, and Xuehai, with the ingredients of Rhizoma Arisaematis, Strychni Semen,Angelicae Dahuricae Radix, and Asari Radix et Rhizoma, 4 h daily, with 15 d as a course of treatment [3]. In addition, acupoint tapping was performed on the hemiplegic side of the patient's limb (the upper limb acupoints were Fengchi, Quchi, and Shuzhe, and the lower limb acupoints were the Zusanli, Yongquan, and Taichong) for 5–10 min each time, two to three times daily [4]. Chinese herbal fumigation was performed on the hemiplegic side of the limb, consisting of Astragali Radix, safflower, Lycopodii Herba, Fistular Onion Stalk (Typhonii Rhizoma was added for phlegm obstruction, and Angelicae Sinensis Radix and Suberect Spatholobus Stem were added for Qi and blood deficiency) for 30 min daily, three times a week.

### 3.1. Observation Indicators

The *Nursing Comfort Rating Scale* developed by our department was used to evaluate the comfort of the two groups of patients before and after the intervention. The scale was scored on three dimensions including physiological comfort, psychological comfort, and hospitalization comfort. The total score is 100 points, and the higher the score, the more comfortable the patient is.

The *Patient Clinical Satisfaction Questionnaire* developed by our department was used to investigate the satisfaction of patients after nursing. The total score on the scale is 100 points. A high score suggests high patient satisfaction. Total nursing satisfaction = satisfied + relatively satisfied.

The *Hospital Anxiety Depression* (*HAD) Scale* [7] was used to assess the emotional state of patients before and after the intervention. The full score of the scale is 42 points. The higher the score, the more severe the anxiety and depression of the patient.

The *Exercise of Self-care Ability Scale* (ESCA) [8] was used to assess the patient's self-care ability. The scale includes self-concept, self-responsibility, self-care skills, and health knowledge, and each item has a total score of 4 points. The higher the value, the better the patient's self-care ability.

*The mini-mental state examination scale* [9] was used to assess the mental state of the patient. The scale has a full score of 30 points. The higher the score, the better the mental state of the patient.

The *BarthelIndex Scale* (BI) [10] was used to assess the patient's self-care ability. The total score on the scale is 100 points. The higher the score, the better the ability of daily living of the patient.

### 3.2. Statistical Analysis

The data analyses were performed using the SPSS20.0 software, and GraphPad Prism 7 (GraphPad Software, San Diego, USA) was used to plot graphics. The count data and measurement data were examined using the chi-square test and *t*-test and normality test, respectively. Statistical significance was set at a *P* value of 0.05 or lower.

## 4. Results

### 4.1. Baseline Patient Profile

The two groups showed similar baseline characteristics such as age, gender, BMI, disease type, smoking, drinking, and place of residence (*P* > 0.05), as shown in Table 1.

### 4.2. Comfort Scores

The experimental group showed higher comfort scores than the control group (*P* > 0.05) (Table 2).

### 4.3. Nursing Satisfaction

The total satisfaction after intervention in the experimental group was higher than that in the control group (*P* > 0.05) (Table 3).

### 4.4. HAD and ESCA Scores

As shown in Figure 1(a), the experimental group had lower HAD scores and higher ESCA scores after intervention than the control group (*P* > 0.05) (Figure 1).

### 4.5. BI Index

The experimental group had a higher BI index after intervention than the control group (*P* > 0.05, Figure 2).

## 5. Discussion

Patients in the *Department of Neurology* are characterized by higher age, acute onset of disease, complex conditions, and a high incidence of risk events [11–13]. Accordingly, the high work intensity of neurology medical staff in nursing care results in a higher chance of nursing errors [14, 15], leading to negative emotions in patients and causing medical disputes. Negative emotions during treatment seriously compromise the prognosis of patients [16, 17]. Comfortable nursing plus psychological nursing is an emerging nursing model and has been clinically recognized. Prior research shows that due to the limited understanding of the disease, neurology patients easily have negative emotions such as anxiety and depression. Comfortable care encompasses the formulation of patient-oriented and reasonable nursing protocols according to the psychological demands of the patients to fulfill the patients' nursing demands for better nursing and treatment efficiency [18–20]. Moreover, psychological care in the treatment of neurology patients scientifically evaluates the patient's mental state and provides them with health knowledge to enrich their understanding of the disease and enhance the treatment compliance. The results of the present study showed that the comfort score of the experimental group after the intervention was significantly higher than that of the control group, indicating that compared with conventional care, comfort care plus psychological care showed a superior effect and satisfied the care needs of patients.

Psychological care promotes patient recovery to alleviate the psychological pressure on the patient [21, 23]. During the nursing period, nurses actively communicate with the patients and provide different psychological support, to effectively lessen the psychological pressure on patients improve the neurological function of patients, and further enrich the improvement of patients' health and ability of daily living [22]. In the current study, comfort nursing plus psychological nursing alleviated the anxiety and depression of patients, indicating a promising nursing outcome of this nursing method. Furthermore, this study showed that the total nursing satisfaction of the experimental group after the intervention was significantly higher than that of the control group, which was consistent with the research results of THUY et al. [23, 24], which revealed that “the nursing satisfaction of the research group (88.24%) was significantly higher than that of 49.02% in the control group,” suggesting that comfort nursing plus psychological care could fulfill the nursing needs of patients, reduce medical disputes, and help create a harmonious nurse-patient relationship. In addition, traditional Chinese medicine care could effectively improve the efficiency of clinical care and the recovery of neurological function of patients, thereby enhancing the quality of life and clinical care of patients. Therefore, the implementation of TCM nursing for patients with cerebral infarction in clinical settings is worth promoting [25].

## 6. Conclusion

Comfort nursing plus psychological care improves nursing satisfaction and self-care ability of neurology patients and relieves their negative emotions.

## Figures and Tables

**Figure 1:** Comparison of HAD and ESCA scores between the two groups (*x* ± *s*) A: the abscissa represents before and after nursing intervention, and the ordinate represents HAD score (points); the HAD scores of patients in the experimental group before and after intervention were (36.11 ± 2.15) points and (4.32 ± 1.05) points, respectively; the HAD scores of the control group before and after intervention were (36.02 ± 2.17) points and (15.11 ± 1.87) points, respectively; the HAD scores of the experimental group patients before and after nursing intervention are significantly different (t = 89.127, ^*∗*^*P* > 0.05). There is a significant difference in the HAD scores of the control group patients before and after the nursing intervention (t = 48.967, ^*∗∗*^*P* > 0.01); there is a significant difference in the HAD scores of the two groups of patients after nursing intervention (t = 33.750, ^*∗∗∗*^*P* < 0.001). B: the abscissa represents before and after nursing intervention, and the ordinate represents ESCA score (points); the ESCA scores of patients in the experimental group before and after nursing intervention were (5.22 ± 0.27) points and (14.89 ± 0.37) points, respectively; the ESCA scores of patients in the control group before and after the nursing intervention were (5.19 ± 0.24) points and (8.36 ± 0.98) points, respectively; the ESCA scores of the experimental group patients before and after nursing intervention are significantly different (*t* = 141.622, ^*∗*^*P* > 0.05); there is a significant difference in the ESCA scores of the control group patients before and after the nursing intervention (*t* = 21.076, ^*∗∗*^*P* > 0.01); the ESCA scores of the two groups of patients after nursing intervention are significantly different (*t* = 41.817, ^*∗∗∗*^*P* < 0.001).

**Figure 2:** Comparison of BI index scores between the two groups (*x* ± *s*). The abscissa represents before and after nursing intervention, and the ordinate represents BI index score (points); the BI index scores of patients in the experimental group before and after nursing intervention were (50.11 ± 2.24) points and (90.11 ± 3.35) points, respectively; the BI index scores of patients in the control group before and after nursing intervention were (50.29 ± 2.21) points and (70.23 ± 3.01) points, respectively; there is a significant difference in the BI index scores in the experimental group before and after nursing intervention (t = 66.584, ^*∗*^*P* > 0.05); there is a significant difference in the BI index scores before and after nursing intervention in the control group (t = 35.821, ^*∗∗*^*P* > 0.01); there is a significant difference in the BI index scores between the two groups of patients after nursing intervention (*t* = 29.612, ^*∗∗∗*^*P* > 0.001).

**Table 1:** Comparison of general information of the two groups of patients.

	Experimental group (*n* = 45)	Control group (*n* = 45)	*x* ^2^/*t*	*P* value
Age (year, *x* ± *s*)			0.086	0.932
	55.75 ± 3.32	55.69 ± 3.29		
Sex (*n* (%))			0.178	0.673
Male	23 (51.11)	21 (46.67)		
Female	22 (48.89)	24 (53.33)		
BMI (kg/m^2^, *x* ± *s*)			1.119	0.266
	26.27 ± 1.59	25.89 ± 1.63		
Disease type (*n* (%))				
Cerebral hemorrhage	21 (46.67)	20 (44.44)	0.045	0.832
Cerebral infarction	10 (22.22)	12 (26.67)	0.241	0.624
Cerebral thrombosis	9 (20.00)	8 (17.78)	0.073	0.788
Smoking [*n* (%)]			0.045	0.832
Yes	20 (44.44)	21 (46.67)		
No	25 (55.56)	24 (53.33)		
Drinking [*n* (%)]			0.178	0.673
Yes	22 (48.89)	24 (53.33)		
No	23 (51.11)	21 (46.67)		
Place of residence (*n* (%))			0.050	0.822
Township	31 (68.89)	30 (66.67)		
Rural area	14 (31.11)	15 (33.33)		

**Table 2:** Comparison of comfort scores between the two groups (*x* ± *s*).

Groups	*n*	Physiological comfort		Psychological comfort		Hospital comfort	
		Before intervention	After intervention	Before intervention	After intervention	Before intervention	After intervention
Experimental group	45	51.35 ± 3.35	91.35 ± 4.27	53.22 ± 3.58	92.36 ± 4.11	55.32 ± 2.36	94.33 ± 3.81
Control group	45	50.88 ± 3.72	72.36 ± 3.98	52.87 ± 3.67	73.25 ± 3.76	54.89 ± 2.93	75.26 ± 3.12
*t*		0.629	21.823	0.458	23.013	0.766	25.977
*P*		0.531	＜0.001	0.648	＜0.001	0.445	＜0.001

**Table 3:** Comparison of nursing satisfaction between the two groups (％ (*n*/*n*)).

Groups	n	Satisfied	Relatively satisfied	Unsatisfied	Total satisfaction
Experimental group	45	68.89% (31/45)	24.44% (11/45)	8.89% (3/45)	93.33% (42/45)
Control group	45	48.89% (22/45)	22.22% (10/45)	28.89% (13/45)	71.11% (32/45)
*x^2^*					7.601
*P* value					＜0.05
